This article has been retracted.

# The influence of environmental factors on seed germination of *Xanthium strumarium* L.: Implications for management

**DOI:** 10.1371/journal.pone.0241601

**Published:** 2020-10-30

**Authors:** Amna Saeed, Ansar Hussain, Muhammad Ifnan Khan, Muhammad Arif, Muhammad Mudassar Maqbool, Hassan Mehmood, Muhammad Iqbal, Jawaher Alkahtani, Mohamed Soliman Elshikh

**Affiliations:** 1 Government Reclamation Research Station, Mian Channu, Pakistan; 2 Department of Plant Breeding and Genetics, Ghazi University, D. G. Khan, Pakistan; 3 Department of Plant Protection, Ghazi University, D. G. Khan, Pakistan; 4 Department of Agronomy, Ghazi University, D. G. Khan, Pakistan; 5 Department of Soil Science, Bahauddin Zakariya University, Multan, Pakistan; 6 Cotton Research Institute, Multan, Pakistan; 7 Department of Botany and Microbiology, College of Science, King Saud University, Riyadh, Saudi Arabia; Harran University, TURKEY

## Abstract

*Xanthium strumarium* L. (Common cocklebur) is a noxious weed prevailing in different ecosystems around the world. It incurs significant yield and economic losses in different cropping systems globally. Successful management of any weed species depends on sound knowledge of seed germination biology. However, detailed knowledge on seed germination biology of the species is missing. Therefore, we investigated the impact of different environmental factors on seed germination and seed burial depths on seedling emergence of two *X*. *strumarium* populations. The impact of different sorghum mulch doses (0–10 t ha^-1^) on seedling emergence of the tested populations was also explored. Seed germination was evaluated under different photoperiods (0, 12 and 24), constant temperatures (0–50°C with 5°C stepwise rise), and different levels of pH (3–12), salinity (0–600 mM) and osmotic potential (0 to -1.6 MPa). Seedling emergence was observed for seeds buried at different depths (0–15 cm). Seeds of both populations proved non-photoblastic; however, higher germination was recorded under 12-hour photoperiod. The seeds germinated under a wide range of constant temperatures (10–45°C), pH (4–10), osmotic potentials (0 to -0.8 MPa) and salinity levels (0–400 mM NaCl). However, the highest germination was observed under 30–31°C temperature and neutral pH (7.51–7.52). Seeds were able to withstand 400 mM salinity and -1.00 MPa osmotic potential. Seedling emergence was initially improved with increasing burial depth and then a sharp decline was noted for the seeds buried >3 cm depth. Most of the seeds of both populations did not emerge from >8 cm depth. Different sorghum mulch doses linearly suppressed seedling emergence of tested populations, and 5.83–5.89 t ha^-1^ mulch application suppressed 50% of seedling emergence. Seedling emergence was completely retarded with 8 t ha^-1^ sorghum mulch. The tested populations germinated under diverse environmental circumstances indicating that the species can become troublesome in marginal habitats and cropped lands. Deep burial of seeds and application of sorghum mulches suppressed seedling emergence. Thus, deep burial followed by shallow tillage and application of sorghum mulches could be used as a successful strategy to manage the species in agricultural fields. Nonetheless, management strategies must be developed to control the species in other habitats.

## Introduction

*Xanthium strumarium* L. (Common cocklebur), a member of the Asteraceae, is an annual weed species propagated by seeds [1, 2]. It is native to North America and Argentina [3], and regarded as a noxious weed species of corn and soybean crops throughout the world [4–8]. Moreover, it produce large amounts of allergenic pollens due to close relatedness of *Xanthium* and *Ambrosia* genus [9–11]. The contact with glandular hairs of the plant causes dermatitis in allergenic individuals [12]. Thus, the species exerts allergenic impact on human population and causes yield and quality losses in different crops.

The infestation of *X*. *strumarium* in cotton caused 5% yield losses in Mississippi, the USA [13]. Similarly, 6–27% cotton yield is lost in North Carolina [14] due to its infestation and critical period of competition is 2–10 weeks after crop emergence [15]. Similarly, groundnut yield is reduced by 31–39% with 0.5 plants m^-2^ density and yield losses may reach ~88% if the density increases to 4 plants m^-2^ [16, 17]. *Xanthium strumarium* infestation in maize causes lower yield losses than in soybean, cotton and groundnut. A 10% reduction in maize yield occurs at 1 plants m^-2^ density and reaches to 27% with 4.7 plants m^-2^ [18]. Nonetheless, it also reduces the yield of horticultural crops [19]. A yield reduction of 5–50% is recorded in snap bean with 0.5 to 8 plants m^-2^ density [20].

*Xanthium strumarium* detrimentally influences livestock production as the animals eating the young plants of species may be poisoned. The young plants of the species are attractive and eaten by the pasture animals. Carboxyatractyloside, a poisoning compound is present in the leaves of young plants of the species, whereas it is not found in older plants [21, 22]. The detrimental impacts of the species on grazing animals have been reported from Australia, where it is frequently noted in pastures [21, 23]. Nonetheless, ‘burrs’ of the species are attached to legs, tails and manes; thus, causing discomfort to the animals.

*Xanthium strumarium* is distributed in several geographic regions of the world and started to exert negative impacts on crop yields, biodiversity and economy [24–27]. Therefore, management strategies are inevitable for the species. The successful management of any weed species depends on the sound knowledge of seed germination biology [28–30]. Seed germination is the first transition step from ‘seed’ to ‘seedling’ in the life cycle of plant species, and readily affected by various environmental factors [31–33]. Nonetheless, seed dormancy level of the seed at different times strongly regulates seed germination of different plant species [34, 35]. Seed germination traits of weed species greatly vary within the same population [36] and among different populations of the same species [28–30]. Seed germination under wide range of environmental conditions guarantees successful establishment and dispersal. Similarly, retarding seed germination or making seeds dormant is the most successful weed management strategy [37]. However, sound knowledge of seed germination biology is essential to manage/suppress weed seed germination.

The seeds of *X*. *strumarium* are rarely dormant, although they possess impermeable seed coat, which becomes permeable soon after seed dispersal. The mature ‘burr’ contains two seed, of which lower one germinates immediately after dispersal (after dry storage for some time), whereas the upper seed remains dormant until the testa is intact [38–42]. More than 80% of the seeds produced by *X*. *strumarium* are viable and exhibit high germination potential [19]. Several studies have investigated the impact of individual environmental factors on seed germination of the species [43, 44]. The seeds are non-photoblastic and do not have strict light requirement for germination [45]. The seeds rarely emerge if buried >15 cm depth [45]. The species requires high moisture for seed germination and rarely emerge if field capacity is <75% [46]. However, the seeds can absorb moisture under increased negative osmotic potential. The seeds lose their viability after few years of dispersal [47]. Although, some information is available on seed germination, the complete knowledge relating to the impact of different environmental factors on seed germination of *X*. *strumarium* is missing.

The use of different mulches has gained increased importance for moisture conservation, weed management and improve soil nutrients [48–52]. The use of plant-based mulches not only lowers cost incurred on crop production, but also solves residue management issue. Nonetheless, mulches did not pose negative impact to crop production; therefore, can be successfully used for weed management [53, 54]. Sorghum [*Sorghum bicolor* (L.) Moench] is an important allelopathic crop and have been reported to suppress seed germination and seedling emergence of several weed species in different crops [55–60]. However, the impact of sorghum mulches on seedling emergence of *X*. *strumarium* has merely been tested.

The current study was conducted to determine the impact of different environmental factors on seed germination of *X*. *strumarium* populations collected from agricultural and ruderal habitats. We were interested to know; i) whether there are differences among seed germination potential of populations stemming from different habitats, ii) are seeds able to germinate under diverse environmental conditions, iii) what is the optimum seed burial depth to retard seedling emergence and iv) what is the optimum dose of sorghum mulch to suppress the seedling emergence of the species. The results of the study would help to develop suitable and effective management strategies against the species.

## Materials and methods

### Site selection and seed collection

The seeds of *Xanthium strumarium* L. populations were collected from Mian Channu. The seeds were collected at maturity, brought to lab, dried under shade (to meet after ripening requirements) and stored at 25°C until use. The seeds were collected from agricultural (30.419203, 72.300121) and ruderal (30.415984, 72.301836) population. Mature ‘burrs’ were collected from 50–60 mother plants. There are no specific permissions required for seed collection and the study did not involve any endangered species. Five laboratory and two greenhouse experiments were conducted to determine the seed germination biology of both populations.

### General experimental procedure

The ‘burrs’ rapidly loose seed dormancy and dormancy release treatments are not required [38, 42]. Therefore, ‘burrs’ of the species were used in the experiments and seeds were not taken off from the ‘burrs’. The 90×15 mm Petri dishes were used to observe seed germination of ‘burrs’ (seeds hereafter). The dishes contained two layers of Whatman no. 1 filter paper, which was moistened with 5 ml deionized water or treatment solution. Paraffin film was used to seal the Petri dishes in order to prevent moisture loss. The dishes were kept at respective environmental conditions for 21 days and then seed germination was observed. There were 20 seeds in one Petri dish and each treatment had five replications. Two Petri dishes were considered as a single replication; thus, each treatment had 10 dishes and 200 seeds. All germination experiments were conducted at 30°C and 12 hours photoperiod with an exceptions for temperature and photoperiod experiments. Seed germination was recorded 21 days after the initiation of the experiments. The non-germinating seeds were tested for viability according to Onen et al. [30] and germination was adjusted for viability. All experiments were terminated after 21 days and repeated over time (two experimental runs for each treatment). The experiments were laid out according to randomized complete block design with split plot arrangement. Populations were regarded as main plot, whereas experimental treatments were randomized in sub-plots.

### Experiment 1: Photoperiod

Seeds were incubated under three different photoperiods (0, 12 and 24 hours) to observe seed germination. The incubators were illuminated with cool, white fluorescent lamps at 380 *μ*Em^−2^ s^−1^ intensity. The dishes of 0-hour photoperiod were wrapped in four layers of aluminum foil for excluding the effects of light.

### Experiment 2: Constant temperatures

Seed germination of both populations was recorded under 10 different constant temperatures (5–50°C with 5°C stepwise increase).

### Experiment 3: pH

Seed germination was noted under 3–11 pH levels. Thus, 10 pH levels were included in the experiment representing, acidic, neutral and alkaline medium. The method of Chauhan et al. [61] was used to prepare solutions of different pH levels.

### Experiment 4: Salinity

Seed germination was recorded under eight different NaCl concentrations (50, 100, 150, 200, 300, 400, 500 and 600 mM). The control treatment (only distilled water) was also included in the experiment for comparison. Sodium chloride (NaCl) was dissolved in distilled water to make the solutions of respective concentrations [28].

### Experiment 5: Osmotic potential

Seed germination of populations stemming from agricultural and ruderal habitats was observed under eight different osmotic potentials (-0.2 to -1.6 MPa), with -0.2 MPa difference among the treatments. The 0 MPa osmotic potential, regarded as control was included in the study for comparison. Polyethylene glycol 6000 was dissolved in distilled water to prepare solutions of respective osmotic potentials [62].

### Experiment 6: Seed burial

The emergence of seeds arising from ruderal and agricultural populations was noted in a pot experiment conducted in greenhouse under controlled conditions. Ten different (0, 0.5, 1, 2, 4, 6, 8, 10, 12 and 15 cm) burial depths were included in the experiment. A total 20 seeds were buried at desired depth. Seedling emergence was recorded 21 days after the initiation of experiment. The pots were irrigated daily to exclude the danger of moisture stress. A mist sprinkler was used to irrigate the pots. The greenhouse was maintained at 30°C and 12-hour photoperiod throughout the experiment.

### Experiment 7: Sorghum mulch

The impact of different doses of sorghum mulch on seedling emergence was recorded in pot experiment. The respective doses were applied at the soil surface after seed sowing. A total 20 seeds were sown in the pots and mulches were applied according to the treatments on soil surface. The greenhouse was maintained at 30°C and 12-hour photoperiod throughout the experiment. The pots were irrigated daily to exclude the danger of moisture stress. A mist sprinkler was used for irrigation. Sorghum plants (above ground parts) were dried to prepare mulches. The dried plants were chopped in a grinding mil to prepare mulches. The resultant powder was regarded as mulch and used according to the treatments.

### Statistical analysis

The final germination percentage data collected were modelled using two different models (sigmoid and Gaussian). The final germination percentage data of osmotic potential, salinity and mulch experiments were modelled by three-parameter sigmd model. The model was

$$G=G_{max}/\left(1+e\;\left[‐x‐T_{50}\right)/G_{rate}\right]$$ (1)

Here; G = seed germination percentage, G_max_ = maximum germination percentage, T_50_ = respective environmental condition for retarding 50% of maximum germination, and G_rate_ = slope.

Similarly, final germination percentage data of temperature, pH and seed burial experiments were analyzed by a three-parameter Gaussian model. The model was:

$$G=a\times e\;\left[‐0.5‐\;{\left\{\left(x-b\right)/c\right\}}^{2}\right]$$ (2)

Here, “a” = the highest seed germination or seedling emergence, “b” = respective environmental condition to achieve the highest germination or seedling emergence and “c” = width of the “bell”. The data of photoperiod experiment were analyzed by two-way analysis of variance (ANOVA) [63]. The homogeneity of variance and normality were tested prior to ANOVA [64]. Least significant difference at 5% probability was used to separate the means. SPSS version 21.0 [65], and SigmaPlot version 13.0 were used for ANOVA and models, respectively.

## Results

### Experiment 1: Photoperiod

Seed germination was influenced by different photoperiods. The seeds of both populations had no strict light requirement for germination, i.e., non-photoblastic. However, higher seed germination percentage was recorded for 12-hour photoperiod compared to 0 and 24-hour photoperiods (Fig 1).

**Fig 1:** The influence of different photoperiods on seed germination percentage of ruderal and agricultural populations of *Xanthium strumarium* L.

### Experiment 2: Constant temperatures

Different constant temperatures strongly mediated the germination of both populations stemming from different habitats. An increase in seed germination percentage was recorded with rise in temperature up to 35°C and then a sharp decline was noted. Agricultural population had higher seed germination (92.66%) compared to ruderal population (81.74%). The highest germination was recorded at 30.62 and 31.08°C for agricultural and ruderal populations, respectively (Fig 2).

**Fig 2:** The influence of different constant temperature regimes on seed germination percentage of ruderal and agricultural populations of *Xanthium strumarium* L.

### Experiment 3: pH

Different pH levels included in the study altered seed germination of populations arising from different habitats. An increase in seed germination was recorded with increasing pH up to 8 and then seed germination sharply declined. Like temperature experiment, agricultural population exhibited higher seed germination (90.64%) compared to ruderal population (85.94%). The highest germination was recorded under 7.51 and 7.52 pH for agricultural and ruderal populations, respectively (Fig 3).

**Fig 3:** The influence of different levels of pH on seed germination percentage of ruderal and agricultural populations of *Xanthium strumarium* L.

### Experiment 4: Salinity

Different salinity levels altered the seed germination of both populations. Seed germination was linearly decreased with increasing salinity level. Overall agricultural population had higher germination ability (95.71%) compared to ruderal population (93.28%). The 50% of the final germination of agricultural population was retarded by 248.55 mM NaCl salinity, whereas 240.56 mM was sufficient to retard 50% of the final seed germination of ruderal population (Fig 4).

**Fig 4:** The influence of different NaCl salinity levels on seed germination percentage of ruderal and agricultural populations of *Xanthium strumarium* L.

### Experiment 5: Osmotic potential

Different osmotic potentials strongly mediated the seed germination of tested populations. A linear reduction in seed germination of both populations was noted with increasing negative osmotic potential. The seeds of agricultural population exhibited higher germination (94.11%) compared to the seeds of ruderal population (87.87%). The osmotic potential required to retard the 50% of the final germination of agricultural population was -0.86 Mpa, whereas -0.87 osmotic potential retarded 50% of the final seed germination of ruderal population (Fig 5).

**Fig 5:** The influence of different osmotic potentials on seed germination percentage of ruderal and agricultural populations of *Xanthium strumarium* L.

### Experiment 6: Seed burial

Different burial depths strongly suppressed the seedling emergence of populations stemming from two distinct. An initial increase was witnessed in seedling emergence up to 3 cm and then a linear reduction was noted. Higher seedling emergence was recorded for agricultural population (82.44%) compared to ruderal population (71.54%). Peak seedling emergence was recorded at 2.88 and 2.87 cm seed burial depths for agricultural and ruderal populations, respectively (Fig 6). Seedling emergence was <20 for the seeds buried at 8 cm depth. Similarly, rare seedling emergences was recorded for the seeds buried >12 cm burial depth.

**Fig 6:** The influence of different seed burial depths on seedling emergence percentage of ruderal and agricultural populations of *Xanthium strumarium* L.

### Experiment 7: Sorghum mulch

The application of different doses of sorghum mulches strongly mediated the seedling emergence of the tested populations. A constant reduction in seedling emergence of both populations was observed with increasing dose of sorghum mulches. Higher seedling emergence was recorded for agricultural population (84.17%) compared to ruderal population (75.78%). The sorghum mulches required to stop 50% of the final seedling emergence percentage were 5.83 and 5.89 t ha^-1^ for agricultural and ruderal populations, respectively (Fig 7). No seedling emergence was noted for >8 t ha^-1^ application of sorghum mulches in both populations.

**Fig 7:** The influence of different sorghum mulch doses on seedling emergence percentage of ruderal and agricultural populations of *Xanthium strumarium* L.

## Discussion

*Xanthium strumarium* populations stemming from different habitats had higher seed germination potential under benign and adverse environmental conditions (Figs 2–5). High germination ability of both populations explain their successful naturalization in different habitats. Furthermore, seed germination ability further warrants range expansion ability to the areas facing different types of abiotic stress, including salinity and drought [28, 30]. Seed dormancy and germination ability are strongly mediated by environmental conditions prevailing during seed set [36, 66]. Seeds of different populations of the same species or even seeds of the same population significantly vary for their seed germination ability [28–30, 36]. These inter and intra-population variations are explained by the adaptive ability and climate prevailing during seed development [36]. Several earlier studies have identified significant variations between different population of the same species for seed germination, growth and fecundity [28–30, 34, 67]. We report that tested populations stemming from different habitats differed in their seed germination ability (Figs 1–5), which is owed to their adaptive ability and environmental conditions faced by maternal plants. The genetic diversity within and among populations might be responsible for these differences; however, this claim needs thorough molecular investigations. The tested populations were able to germinate under diverse environments (Figs 1–5), indicating that both populations have a wide seed germination niche. There are several earlier studies indicating that weed species possess a broad seed germination niche, which help them to adapt stressful and benign environments [28–30, 68].

Photoperiod had a slight impact on seed germination of tested populations. The seeds proved non-photoblastic; however, higher seed germination was noted for 12-hour photoperiod. The results are in line with Weaver and Lechowicz [19] who reported that seed germination of *X*. *strumarium* did not depend on light availability. Overall, ruderal population exhibited low germination than agricultural population, which can be attributed to the disturbance faced by agricultural population. The seeds of ruderal population did not face frequent disturbance; thus, are less tolerant to adverse environmental conditions.

Seed germination is strongly dependent on soil temperature since numerous enzyme activities are regulated by temperature [31, 69]. The tested populations exhibited seed germination under almost all tested temperatures with little differences. The optimum temperature ranged from 31 to 32°C for agricultural and ruderal populations. The earlier findings have also indicated that optimum temperature for seed germination of *X*. *strumarium* is 30–35°C [43, 44]. There were slight differences among tested populations for optimum temperature requirement. The differences in seed traits of different species due to selection in different environments have been explained earlier [70, 71].

The establishment of plant species is strongly obstructed by salinity, pH and water stress. Germination ability under diverse pH, salinity and water stress levels guarantees the persistence and establishment of weed species [72]. The tested populations were able to germinate under diverse pH, salinity and osmotic potential levels. The germination of the tested populations under elevated pH, salinity and osmotic potential levels indicate that species could establish and persist in marginal habitats.

Seedling emergence increased up to 3 cm and followed by a sharp decline under deeper seed burials. The low emergence of the surface placed seeds can be linked to poor soil-seed contact and less water imbibition [33]. Seeds were able to emerge even form 8 cm seed burial depth. The emergence from deeper soil layers helps the species to persist in soil seed bank for longer time [73]. Several studies have reported that deep burial of the seeds of various weed species significantly decreased or even halted their seedling emergence [28–30, 32]. It seems that burying seeds to maximum depth of emergence could combat the species agricultural habitats. However, topsoil is turned over by moldboard plow (conventional tillage) which help the seeds to included in the seed bank again. The weed management strategy must focus on decreasing seedling emergence, seed production and addition of seeds to soil seed bank. This will progressively reduce soil seed bank. Shallow tillage and management of the emerging seedlings through integrated weed management approach seems a viable option for the management of the species.

The use of different mulches is becoming popular in wake of sustainable agriculture [50, 51, 58]. Sorghum mulches have been successfully used to suppress the germination and growth of several weed species [56, 57, 60]. The applied mulched significantly reduced seedling emergence of the populations included in the study. Thus, deep burial, shallow tillage and application of sorghum mulches could be successfully used to manage the species in agricultural habitats.

## Conclusion

The tested populations germinated under diverse environmental conditions, which indicates that the species can become noxious in marginal and cropped lands. The deep burial of seeds and application of mulches suppressed seedling emergence of the species. Thus, deep burial, shallow tillage and application of sorghum mulches could be successfully used to manage the species in agricultural habitats.
